The article "Ethnobotanical study of traditional medicinal plants in Kebridehar and Shekosh districts, Korahi zone, Somali Region, Ethiopia" was retracted in 2025. Reasons: lack of ethics approval or compliance; concerns about the welfare of human subjects.

# Ethnobotanical study of traditional medicinal plants in Kebridehar and Shekosh districts, Korahi zone, Somali Region, Ethiopia

**DOI:** 10.1016/j.heliyon.2023.e22152

**Published:** 2023-11-19

**Authors:** Kassaw Awoke Wubu, Ayichesh Haymiro Ngatie, Tilaye Aregu Haylie, Abdikader Dekane Osman

**Affiliations:** Kebridehar University, Department of Biology, P.O. Box 250, Ethiopia

**Keywords:** Ethnobotanical, Antibacterial, Traditional healer, Medicinal plant, Kebridehar, Shekosh

## Abstract

This study was conducted in Kebridehar and Shekosh districts, Ethiopia, to investigate an ethnobotanical study on traditional medicinal plants. Systematic random sampling techniques were used for data collection. Preference ranking, paired comparison, informant consensus factor, direct matrix ranking, and jaccard comparison were used for data analysis. A total of 44 medicinal plant species from 34 genera and 23 families have been documented as being used to treat 38 human, 5 livestock, and 1 both human and livestock ailment. The shrub category was the dominant growth form in the study area. The study showed that the most frequently used plant parts for the preparation of traditional medicine were roots (45.45 %), followed by leaves, glue, and liquid (11.36 % each). The most common route of administration was oral (30.77 %), followed by dermal (20.51 %). Jaccard's Coefficient of Similarity for Kebridehar and Shekosh for the reported traditional medicinal plants were 0.21, indicating some trend towards using common plants. Methanol extracts were more effective than ethanol extracts. The results of this study provide an insight into the anti-bacterial properties of the extracts of Aloe megalacantha, Ephorbiarobecchi, and Oppiliacampestris. This in vitro study demonstrated that these three folklore medicinal plants have good potential. In conclusion, the main threat to medicinal plants in the study area was drought. Therefore, it is recommended that the cultivation of medicinal plants be encouraged in home gardens.

## 1 Introduction

Ethnobotany is the study of how local people interact with the natural environment: how they classify, manage, and use the plants that are available to them [1]. The documentation of traditional medicinal plant applications is a pressing issue that must be addressed in order to preserve knowledge [2].

In developing countries, up to 80 % of populations depend on plants for their primary healthcare [3], and the value of medicinal plants to human livelihoods is essentially infinite [4]. According to Ref. [5], the current loss of medicinal plants in the nation as a result of anthropogenic and natural processes is connected with the loss of priceless indigenous knowledge related to the plants. As a result, indigenous knowledge is vanishing and plant resources are being exhausted more quickly. As in many other regions of Ethiopia, this issue was discovered in the districts of Kebridhar and Shekosh. The objectives of the present study were: a) to identify plant species used for medicinal purposes in treating human and livestock health problems in the study area; b) to collect, record, and document indigenous knowledge of the people on medicinal plants in the study area; c) to identify plant parts used to treat diseases, method of preparation, and route of administration as used by the local people in the study area; d) to assess the role of traditional practices and indigenous knowledge in maintaining medically important plant species; e) to find out the threats and local methods used by the indigenous people to conserve medicinal plants; and f) to identify the antibacterial activity of some selected medicinal plants against pathogenic bacteria.

The article "Ethnobotanical study of traditional medicinal plants in Kebridehar and Shekosh districts, Korahi zone, Somali Region, Ethiopia" was retracted in 2025. Reasons: lack of ethics approval or compliance; concerns about the welfare of human subjects.

## 2 Materials and methods

### 2.1 Reconnaissance survey and selection of study sites

A reconnaissance survey of the study area was carried out from January 2 to 21, 2021. The study locations were chosen based on recommendations with the assistance of local officials, elders, and altitudinal range. Consequently, sixkebeles from various agro-climatic zones participated in the study.

### 2.2 Description of the study area

The study was carried out in two districts of the Somali regional states of Kebridehar and Shekosh in the Korahie Zone. Ethiopia's capital city, Addis Ababa, is 1004 km away. Between 6° 28′–7° 68′ N latitude and 43° 53′–45° 00′ E longitude and 6° 78′–7° 6′ N latitude and 43° 54′–44° 49′ E longitude, respectively, were the Kebridehar and Shekosh districts (Fig. 1).

**Fig. 1:** Map of the study area.

The districts of Kebridehar and Shekosh are situated in Ethiopia's southeast lowlands, at an altitude of 456 and 1042 m above sea level, respectively. The mean annual temperature varies from 20.75 °C to 31.25 °C, with high temperatures and little precipitation being experienced in a substantial section of both districts. The annual rainfall in the districts ranges from 295 mm to 595.6 mm.

### 2.3 Informant selection

As a result, a total of 74 informants (37 male and 37 female) ranging in age from 15 to 80 were chosen purposefully and randomly from the representative group of kebele informants. On the advice of the local authorities, kebele agricultural officials, knowledgeable elders, religious leaders, and members of the local community, key informants were purposefully chosen from the study location. On the advice of knowledgeable elders, responsible locals, and development professionals, 24 essential key informants were purposefully chosen. The quality of the justifications given by specific interviews during the selection of significant participants was also taken into account. Local healers were automatically certified as key participants as traditional experts who are stewards of indigenous knowledge about medicinal herbs [1].

The article "Ethnobotanical study of traditional medicinal plants in Kebridehar and Shekosh districts, Korahi zone, Somali Region, Ethiopia" was retracted in 2025. Reasons: lack of ethics approval or compliance; concerns about the welfare of human subjects.

### 2.4 Semi-structured interview

Eleven main questions were prepared for a semi-structured list that was discussed in a specific order with the informants (Appendix 1). All responses were recorded in English, and all interviews were conducted in Afan Somali, which is the local tongue spoken most frequently by the informants. Each informant's interview was conducted separately. It involved people who were either born in the area or had spent the majority of their lives there. Information about the local name of the medicinal plant, the health issues treated, the parts used, the preparation methods, the mode of application, the ingredients used in combination, threats and management, and other pertinent ones were noted during the interview [6].

### 2.5 Guided field walk

The study included a field walk with guides and/or traditional healer(s), as recommended by the research [1,5]. All necessary data, including the common and scientific names of plants, the parts used, the preparation methods and administration routes, the diseases to be treated, and their cultural knowledge for the conservation and preservation of medicinal plants, were gathered during the guided field walk.

### 2.6 Group discussion

Focus groups were held to verify the authenticity of the information acquired through semi-structured interviews and to gain greater insight into local knowledge of medicinal plants [1]. One focus group meeting per of the six kebeles in the district was held. There were five to seven informants per kebele, and traditional healers occasionally joined the discussion to provide some of the common traditional wisdom with the informants selected for it.

### 2.7 Data collection

A letter of agreement was given by Kabridahar University before the data gathering got started. To obtain verbal consent from the participants, group talks on the study's objectives were held prior to the interviews. All participants provided oral consent, and this consent was used to gather all of the data.

Ethnobotanical information was acquired from February through May 2021. Conventional data collection methods have been used to capture the local community's traditional knowledge of health, the usage of medicinal plants, conservation initiatives, and hazards [1]. For ethnobotanical research, semi-structured interviews, field observations, guided field walks, market surveys, and group discussions were employed as data gathering methods. Semi-structured interviews were conducted using a list of questions that had been created in English and translated into “Somali,” the language of the region. During an interview with a participant, information was meticulously recorded. The important points on the checklist were covered during the interview under guidance. Based on the participants' level of interest, the interview location and time were chosen. The morphological characteristics and habitats of each species of medicinal plant were observed in the field with the assistance of local guides. The therapeutic plants in the study region were briefly discussed in groups with the participants.

The article "Ethnobotanical study of traditional medicinal plants in Kebridehar and Shekosh districts, Korahi zone, Somali Region, Ethiopia" was retracted in 2025. Reasons: lack of ethics approval or compliance; concerns about the welfare of human subjects.

Threats to medicinal plants, their preservation, and the sharing of information within the community were all discussed. The plant parts were cleaned with tap water, dried outside, and ground to the appropriate size before extraction [7]. The postgraduate microbiology lab at Bahir Dar University ran a lab experiment in June–July 2021 to investigate the antibacterial activity of various selected plant species extracts against various dangerous bacteria.

### 2.8 Specimen collection and identification

Locally collected medicinal plants were counted, pressed, and dried for identification while on a guided field trip. The specimens were identified in the herbarium and in the field. Using taxonomic keys, experts, and various books on Ethiopian and Eritrean flora, the plants were identified between May and June.

### 2.9 Extraction of plant materials

Plant material was extracted by macerating it for three days at room temperature with methanol and ethanol solvents while shaking it occasionally. Separately, the extracts were concentrated in a dry oven at 80 °C for 4 h after being filtered through Whatman No. 1 filter paper [8].

### 2.10 Antibacterial activities of selected plant part extracts

#### 2.10.1 Source of the test bacterial pathogens and inoculum preparation

In addition to clinical isolates of bacteria, the Bahir Dar Public Health Institute also offered representative gram-negative and gram-positive bacteria (standard reference). The bacteria employed in the study were produced by inoculating isolates into nutritious broth and culturing them at 37 °C for 24 h. The culture turbidity was adjusted to a McFarland standard of 0.5 using sterile normal saline [7].

#### 2.10.2 The antibacterial assays

The agar-well diffusion method was used to test the antibacterial activity of the crude extracts of three plant species against bacteria. Using sterile cotton swabs previously produced standardized bacterial broth cultures were swabbed on Mueller-Hinton Agar (Himedia) plates. A 6 mm-diameter sterilized corkborer will be used to drill five evenly spaced wells on each plate after 30 min [7]. Stock solutions of each plant extract were made using sterilized distilled water at various concentrations (25, 50, and 100 mg/ml), and 100 l of each plant extract were aseptically added to the wells. The plates were incubated in triplicates for 18–24 h at 37 °C after being allowed to diffuse at room temperature for 2 h. Gentamicin (0.01 mg/ml) was employed as a positive control and sterile distilled water without plant extract as a negative control, respectively. By using a ruler to measure the diameter of the zone of inhibition in mm, the antibacterial activity was assessed [7].

The article "Ethnobotanical study of traditional medicinal plants in Kebridehar and Shekosh districts, Korahi zone, Somali Region, Ethiopia" was retracted in 2025. Reasons: lack of ethics approval or compliance; concerns about the welfare of human subjects.

### 2.11 Determination of minimum inhibitory concentration and minimum bactericidal concentration

The two-fold broth dilution method for calculating the minimum inhibitory concentration (MIC) of extracts demonstrated significant antibacterial activity when compared to the agar-well diffusion methodology [7]. The plant extract solutions (100 mg/ml) were serial dilution with nutrient broth as 1:2, 1:4, 1:8, 1:16, 1:32, 1:64, 1:128 and 1:256 to bring 50 mg/ml, 25 mg/ml, 12.5 mg/ml, 6.25 mg/ml, 3.125 mg/ml, 1.56 mg/ml, 0.78 mg/ml and 0.39 mg/ml concentrations, respectively and 20 μl of a standard suspension of test organisms were added to each concentration of the extract. Extra test tubes containing peptone water and peptone water plus the test organisms were prepared to serve as a negative and positive control, respectively [8]. The broth tubes were incubated at 37 °C for 24 h. The lowest concentration in the test tube that didn't cause any growth or turbidity was identified as the extract's MIC value. The MBC value against the tested bacterial species was calculated using the lowest concentration of the tested extracts that displayed no detectable growth during incubation [9].

A loop full of inoculums was streaked on nutritional agar plates from all the tubes that did not exhibit any visible evidence of growth or turbidity (100, 50, 25, 12.5, 6.25, 3.125, and 1.56 mg/ml). These plates were then incubated at 37 °C for 24 h. The MBC value of the tested extracts against the tested bacterial species will be determined by the lowest dose at which there was no discernible growth during incubation [7].

### 2.12 Data analysis

[1,2], and [6] assert that the ratios of growth habit, plant part(s) employed, medicinal plant condition, method of administration, preference ranking, paired comparison, informant consensus, and direct matrix ranking were computed using Microsoft Excel software. With the aid of SPSS, the minimal inhibitory concentration, minimal bactericidal concentration, and antibacterial properties of the selected plant extracts were determined.

The article "Ethnobotanical study of traditional medicinal plants in Kebridehar and Shekosh districts, Korahi zone, Somali Region, Ethiopia" was retracted in 2025. Reasons: lack of ethics approval or compliance; concerns about the welfare of human subjects.

### 2.13 Informant consensus

Informants were questioned at least twice about the same ideas in order to assess the reliability of the information given during the interview. The information's reliability was confirmed and noted. As a result, if the informant's proposal differs from the initial information, it is rejected since it is thought to be unreliable. Therefore, only those that were relevant were considered and statistically analyzed. This method is based on the [1] formula. $\text{ICF}=\frac{n\text{ur}-\text{nt}}{nur-1}$.

### 2.14 Preference ranking

Preference ranking was one of the previously designed items for a semi-structured interview. According to Ref. [5], a preference assessment is conducted for the six most important medicinal plants used to treat an illness as it is treated by traditional healers. The key informants were selected to determine the most highly recommended medicinal plants for the treatment of ailments based on their personal preferences or perceived level of relevance in the community. Each informant received a report on six medicinal plants that could be used to treat ulcers. Participants were asked to rank the remaining plants from least to most effective against this ailment, with one being the least effective and six being the highest. The names of the medicinal plants were inscribed on the leaves. The data was then added together, put in a certain order, and displayed in tables.

### 2.15 Direct matrix ranking

According to Refs. [1,6], direct matrix ranking is employed. Each key informant assigned things after carefully weighing various characteristics one at a time. A numerical scale was used, with the greatest number being the most preferred item and the lowest number representing the least preferred one. The respondents ranked their favorites out of six. Direct matrix ranking can also be done in a group setting where participants agree on the order of each item or cast their votes individually [5]. Based on the information received from informants, six multipurpose tree species were selected from the total medicinal plants, and seven use varieties of these plants were listed for six key informants to assign use values to each species. One or more of the seven use values include medical, food, firewood, building, charcoal, fencing, and furniture manufacturing. The values of each species were then totaled up and sorted, and the average value of each species' many uses was determined.

The article "Ethnobotanical study of traditional medicinal plants in Kebridehar and Shekosh districts, Korahi zone, Somali Region, Ethiopia" was retracted in 2025. Reasons: lack of ethics approval or compliance; concerns about the welfare of human subjects.

### 2.16 Paired comparison

Five different types of medicinal plants are used to treat fibril illness, and [1] presented paired comparisons to demonstrate their acceptance and effectiveness, along with six significant informants. The order of the pairings and the components within each pair were both randomized after, and a list of all possible pairings of the provided elements was created. The pairs were then presented to the chosen informants, and their comments were noted. The sum of all scores was calculated using the formula n (n-1)/2, where n is the total number of medicinal plants taken into account.

### 2.17 Jaccard’s Coefficient of similarity

Using Jaccard's Coefficient of Similarity, it was possible to compare the species composition of several districts (JCS). It is determined by comparing the study areas to other locations that have been the focus of studies carried out by other writers in various regions of the nation [1]. calculated JCS as follows: JCS $=\frac{c}{\left(a+b+c\right)}$.

### 2.18 Analysis of antibacterial activity

One-way analysis of variance and Duncan's multiple comparison tests were used to examine the statistical differences in the mean zone of inhibition, MIC, and MBC of extracts for each bacterium and among bacteria using the Statistical Package for the Social Sciences (SPSS) Version 20 software [7]. The data obtained from the experiments were analyzed carefully by calculating their mean of triplicate and standarddeviationsto determine whether there was significant difference in zone of inhibition between extracts concentrations. A *P*-value of less than 0.05 was used to indicate statistical significance.

## 3 Ethical consideration

The Kebridehar University member institution's Ethics Committee gave its approval for this project. The goal of the study was explained to the participants, who completed the questionnaire in an anonymous manner while having the option to skip any questions they did not wish to answer. The dignity of research participants should be respected, and prior to the study, participants' full agreement should be sought. Moreover, the confidentiality of research participants' personal information must be protected. Ethical consent was approved by GebeyehuAmare, TeklayGebru, and Belayneh Daniel, who are affiliated with Kebridehar University.

## 4 Result

### 4.1 Information about the informants in the study area

#### 4.1.1 Ages of informants

The majority of knowledgeable elders are between the ages of 51 and 65, according to the age distribution of informants (Table 1). This indicates that most traditional healers agreed that there were no restrictions on harvesting and using medicinal plants in the study region. The ages of the healers and the number of medicinal species reported by each traditional healer were strongly correlated. Traditional healers who were older than those who were younger cited more medicinal plant species.

The article "Ethnobotanical study of traditional medicinal plants in Kebridehar and Shekosh districts, Korahi zone, Somali Region, Ethiopia" was retracted in 2025. Reasons: lack of ethics approval or compliance; concerns about the welfare of human subjects.

**Table 1:** Ages of informants in the study area.

Informant age	No. of informants	Percent
20–30	12	16.22 %
31–40	15	20.27 %
41–50	22	29.73 %
51–65	25	33.78 %

#### 4.1.2 Marital status of informants in study area

Despite the fact that 79.73 % of all informants were married, just 16.22 % and 4.05 % of them were single or divorced, respectively (Table 2). The relationship between each informant's reported number of medicinal species and their marital status was crucial. More medicinal plant species were mentioned by married interviewees than by single or divorced interviewees.

**Table 2:** Marital status of informants.

	Sex		Total	Percentage
Maritalstatus	F	M		
Married	26	33	59	79.73 %
Single	6	6	12	16.22 %
Divorced	3		3	4.05
Total	35	39	74	100

#### 4.1.3 Educational status of informants

The informants in the study had a variety of educational backgrounds, including religious education, grades eight through twelve of a diploma or certificate program, and illiteracy. Religious education ranked first with 39.19 %. Illiteracy came in second with 36.49 % of the total, followed by other variables with 24.33 % (Table 3). This indicates that there is a poor correlation between the informants' present level of education and their familiarity with ethnobotany. As one's academic standing increases, their knowledge of ethnobotany decreases.

**Table 3:** Educational status of informants.

Educational status	Grade	Percentage
Illiterate	27	36.49 %
Writing and reading	10	13.51 %
8–12	4	5.41 %
Diploma and certificate	4	5.41 %
Religious education	29	39.19 %
Total	74	100.00 %

### 4.2 Medicinal plants of the study area

Several plant species are used by locals in the study area for traditional medical purposes, including the treatment of human and animal ailments. From the research region, 44 plant species were gathered and divided into 34 genera and 23 families. With nine species, the Fabaceae family has the most diversity, followed by Burseraceae, Euphorbiaceae, and Solanaceae, each of which has four species (Fig. 2).

**Fig. 2:** Number of medicinal plants in each family.

### 4.3 Habits of medicinal plants

The most prevalent growth forms of these medicinal plants are shrubs, with 25 (56.82 %) species, trees with 10 (22.73 %) species, herbs, with 8 (18.18 %) species, and lianas, with 2 (4.55 %) species, according to an analysis of their growth forms (Fig. 3).

**Fig. 3:** Habits of medicinal plants.

Medicinal Plants Used to Treat Human, Livestock, and Both Human and Livestock Ailments in the Study Area.

The article "Ethnobotanical study of traditional medicinal plants in Kebridehar and Shekosh districts, Korahi zone, Somali Region, Ethiopia" was retracted in 2025. Reasons: lack of ethics approval or compliance; concerns about the welfare of human subjects.

The study area's data revealed that 38 (86.36 %), 5 (11.36 %), and 1 (2.27 %) medicinal plants were used, respectively, to cure only human, livestock, and human and animal disorders.

### 4.4 Parts of Medicinal Plants Used to Treat Human and Livestock Ailments

Parts of medicinal plants are used to treat human ailments.

In the Kebridehar and Shekosh districts of the research area, 38 plant species were utilized to cure 52 human diseases, with roots alone accounting for 19 (50 %) of the cases and leaves for 4 (10.53 %) (Fig. 4).

**Fig. 4:** Plant parts used to treat human ailments.

Parts of medicinal plants are used to treat livestock ailments.

In the Kebridehar and Shekosh districts of the research area, six cattle ailments were treated with the help of five plant species: liquids accounted for the bulk of cases (40.00 %), followed by leaves, cork, and root, each of which accounted for 20.00 % of the cases (Table 4).

**Table 4:** Plant parts used to treat livestock ailments.

Plant Parts used	No. of species	%
Leaves	1	20.00 %
Root	1	20.00 %
Liquid	2	40.00 %
Cork	1	20.00 %

### 4.5 Mode of preparation used to Treat Human and Livestock Ailments

Mode of preparation used to treat human ailments.

The indigenous inhabitants prepare traditional remedies using a variety of methods to cure a range of ailments. Different preparations are used depending on the type and location of the illness. According to reports, the bulk of the plant materials used to make remedies were crushed into a powder and used for 10 (26.32 %) of the plant materials. The next most popular techniques were crushing 6 (15.79 %), harvesting glue 4 (10.53 %), crushing boiling 4 (10.53 %), and harvesting liquid 3 (7.89 %). The remaining components are produced by a variety of processes, including mixing, boiling, chewing, making decoctions, burning, foaming powder, harvesting fluids, and combining (Fig. 5).

**Fig. 5:** Mode of preparation for human ailments.

Mode of preparation used to treat livestock ailments.

Depending on the condition being treated and local expertise, the preparations vary. The most popular way to prepare plant part remedies was reported to be harvest liquid, which accounted for 2 (40 %), followed by crushing, dizzying, and crushing with bite, each of which accounted for 1 (20 %) (Fig. 6).

**Fig. 6:** Methods of preparation for livestock ailments.

### 4.6 Mode of administration used to Treat Human and Livestock Ailments

Mode of administration used to treat human ailments.

The most common method of administration was oral, accounting for 11 (28.95 %) of all occurrences, followed by dermal, accounting for 8 (21.05 %) of all occurrences (Fig. 7).

The article "Ethnobotanical study of traditional medicinal plants in Kebridehar and Shekosh districts, Korahi zone, Somali Region, Ethiopia" was retracted in 2025. Reasons: lack of ethics approval or compliance; concerns about the welfare of human subjects.

**Fig. 7:** Mode of administration for human ailments Mode of administration used to treat livestock ailments.

In the research area, dermal administration was used 3 times (60 %) while oral and biting-pouring administration w*ere used 1* time (20 %) (see Fig. 8).

**Fig. 8:** Mode of administration used to treat livestock ailments.

### 4.7 Ranking of important medicinal plants

#### 4.7.1 Preference ranking

People prefer one species over another when several are suggested for the same health issue. In the preference rating exercise carried out by Ref. [5], six key informants ranked six medicinal plants that have been proposed as ulcer treatments. According to the informants' rankings of the medicinal plants' efficacy in treating ulcers, *Lyciumshawii* was found to be the least useful and *Euphorbia robecchii* to be the most helpful (Table 5).

**Table 5:** Preference ranking of medicinal plants used for treating ulcers.

	Informants							
List of medicinal plants	I1	I2	I3	I4	I5	I6	Total	Rank
*Euphorbia robecchii*	6	5	6	5	5	6	33	1
*Grewiatenax*	5	3	2	4	6	2	22	4
*Hydnorajohanni*	2	6	5	2	3	2	20	5
*Lyciumshawii*	2	3	4	2	2	5	18	6
*Ricinuscommunis*	4	4	3	5	4	4	24	3
*Desmodiummolliculum*	4	3	5	6	4	4	26	2

Key: I= Informants.

#### 4.7.2 Paired comparison

The informants identified medicinal herbs that may be used to treat stomach ailments, the most common illness for which people seek out traditional healers rather than modern institutions. Pair-by-pair comparisons were done by five of them (Table 6).

**Table 6:** Paired-wise comparison of medicinal plants used for gastric.

	Informants							
Medicinal plants	I1	I2	I3	I4	I5	I6	Score	Rank
*Acacia Senegal*	3	5	4	5	4	5	26	1
*Aloe megalacantha*	5	4	3	2	4	4	20	2
*Blepharisedulis*	2	2	5	3	2	1	15	5
*Commiphoraguidottii*	1	3	3	3	5	2	17	4
*Moringastenopetala*	4	2	4	4	2	3	19	3

Key: I = Informants.

#### 4.7.3 Direct matrix ranking

Other than for medical purposes, a number of medicinal plants have been used for a variety of purposes. The most often used applications include those for food, fuel, construction, charcoal, fencing, and agricultural equipment. The six key informants gave the most frequently used plant for that purpose a score of five, while giving the least frequently used species a score of zero. The most adaptable plants were also found to be *Acacia senegal*, *Acacia tortilis*, and *Balanitesglabra*, with a total score of 148 for *Acacia senegal,* 140 for *Acacia tortilis*, and 67 for *Balanitesglabra* (Table 7).

**Table 7:** Direct matrix ranking for the multipurpose of five medicinal plants:The value given to each plant is the sum of the scores given by the informants.

	Name of the Species					
Use category	*Acacia mellifera*	*Azadirachtaindica*	*Boswelliarivae*	*Acacia tortilis*	*Acacia senegal*	*Balanitesglabra*
Medicinal	26	20	19	25	22	15
Food	25	19	20	23	18	13
Fire wood	21	10	15	20	26	10
Construction	21	11	11	20	23	5
Charcoal	13	6	11	21	20	6
Feancing	15	14	14	16	19	13
Agricultural tool	13	12	10	15	20	5
Total	134	92	100	140	148	67
Rank	3	5	4	2	1	6

The article "Ethnobotanical study of traditional medicinal plants in Kebridehar and Shekosh districts, Korahi zone, Somali Region, Ethiopia" was retracted in 2025. Reasons: lack of ethics approval or compliance; concerns about the welfare of human subjects.

#### 4.7.4 Informant consensus

An examination of informant consensus showed that some therapeutic plants were more popular than others. Twelve people (16.21 %) mentioned *Solanumincanum*, whereas ten people (13.51 %) mentioned *Euphorbia schizocantha* (Table 8).

**Table 8:** Informant consensus of medicinal plants in the study area.

Scientific name	No. of informants cited	%	Rank
*Acacia Senegal*	3	4.05 %	8
*Blepharisedulis*	2	2.7 %	9
*Commiphoraguidotti*	8	10.81 %	4
*Commiphoramyrra*	7	9.45 %	5
*Cucumispustulatus*	4	5.4 %	7
*Euphorbia schizocantha*	10	13.51 %	2
*Grewia* spp.	9	12.16 %	3
*Moringastenopetala*	5	6.75	6
*Solanumincanum*	12	16.21 %	1

#### 4.7.5 Informant consensus factor (ICF)

The findings demonstrate that specific medicinal plants are useful in treating particular illnesses. The diseases in the research area have been categorized into different groups based on the region where the disease is most prevalent, its severity, and how similar the condition's treatment is to that of the local population. For each category, the informant consensus factors have been determined (Table 9).

**Table 9:** Informant consensus factor (ICF).

Human disease category	Nt	% of Nt	Nur	% of Nur	ICF	%ICF
Malaria and Fever	3	11.54	19	14.07	0.88	88
Hemorrhoid& Cardiovascular	7	26.92	38	28.15	0.84	84
Diarrhea&Typhoid	3	11.54	13	9.63	0.83	83
Ulcers& Skin diseases	7	26.92	26	100	0.76	76
Stomach gastric	4	15.38	35	100	0.91	91
Fertility & maternal	2	7.69	4	2.93	0.67	67

#### 4.7.6 Fidelity level of medicinal plants

The FL results in this investigation ranged from 25 % to 100 %. The only known plant species with a faithfulness level of 100 % are *Acacia senegal, Blepharisedulis*, and *Opoiliacampestris*; all other species have a fidelity rating of less than 100 % (Table 10). The most prevalent species, *Commiphoramyrrha*, which is believed to treat a number of illnesses, was found to only have a FL value of 25 %.

**Table 10:** Fidelity level index of the most commonly used medicinal plants.

Species	Ailment treated	Ip	Iu	FL	FL%
*Acacia Senegal*	Gastric	7	7	1	100
*Blepharisedulis*	Tooth, gastric, obstruction urine	1	1	1	100
*Opoiliacampestris*	Common cold/Influenza	1	1	1	100
*Acacia tortilis*	Increase eye sitting	8	9	0.89	89
*Coleus barbatus*	Headache	6	7	0.86	86
*Otostegia modest*	Paralysis	6	7	0.86	86
*Commiphoraguidotti*	Gastric, remove after delivery	6	7	0.86	86
*Ricinuscommunis*	Ulcers	2	7	0.29	29
*Commiphora myrrh*	Swelling	1	4	0.25	25

The article "Ethnobotanical study of traditional medicinal plants in Kebridehar and Shekosh districts, Korahi zone, Somali Region, Ethiopia" was retracted in 2025. Reasons: lack of ethics approval or compliance; concerns about the welfare of human subjects.

#### 4.7.7 Jaccard coefficient of similarity

The study conducted in Southwest Oromo had the highest degree of resemblance, followed by the current study (20.8 %), and then Wonagowereda (19.3 %), according to the comparison's findings using the Jaccard coefficient of similarity (Table 11).

**Table 11:** The Jaccard coefficient similarity in the study area with two other areas with respect to medicinal plant composition.

Sample area	A	B	C	%JCS	Source
Kebridehar&shekosh	40	36	20	20.8	This study
WonagoWereda	58	29	29	19.3	[10]
Southwest Oromo	67	34	33	21.2	[11]

### 4.8 Threats from medicinal plants in the study area

#### 4.8.1 Factors threatening medicinal plants

The most significant hazard to medicinal plants in the study area is firewood, followed by drought and charcoal collection, whereas overgrazing is a less major threat (Table 12).

**Table 12:** Ranking of threats to medicinal plants.

Threats	R1	R2	R3	R4	R5	Total	Rank
Drought	3	4	4	4	3	18	2
Fire wood	3	4	4	5	5	21	1
Charcoal	3	4	3	2	4	16	3
Construction	2	3	3	1	4	13	4
Overgrazing	2	1	4	2	3	12	5

### 4.9 Activities on gram-negative and gram-positive bacteria

The antibacterial activity of three plant species against gram-positive and gram-negative bacteria using the agar diffusion method is shown in Table 13 at 25, 50, and 100 mg/ml test concentrations with methanol extract, and it is shown in Table 14 at 25, 50, and 100 mg/ml test concentrations with ethanol extract. The antibacterial activity of methanol extracts from the three plants against gram-positive bacteria was determined using the agar-well diffusion assay, the results of which are shown in Table 13.

**Table 13:** Antibacterial activity of three selected plantswith methanol extracts against gram-positive and gram-negative bacteria using the well diffusion method.

Plant species	Concentration	Inhibition zone of methanol extract Diameter (mm) (Mean ± S.D)	
		E.coli	S.aures
*Euphorbia robecchi*	25	11.00 ± 0.58	10.67 ± 0.33
	50	15.00 ± 0.00	18.00 ± 0.00
	100	18.00 ± 0.00	13.67 ± 0.33
*Aloe megalacantha*	25	15.33 ± 0.33	11.33 ± 0.67
	50	17.00 ± 0.00	15.00 ± 0.00
	100	20.00 ± 0.00	16.00 ± 0.00
*Opoiliacampestris*	25	7.33 ± 0.33	7.67 ± 0.33
	50	8.67 ± 0.33	8.00 ± 0.58
	100	9.33 ± 0.33	9.00 ± 0.58
Tetracycline	Sta.	22.00 ± 0.00	22.00 ± 0.00

Values are expressed as the mean of three replicates ± standard deviation.

**Table 14:** Antibacterial activity of three selected plantswith ethanol extracts against gram-positive and gram-negative bacteria using the well diffusion method.

Plant species	Concentration	Inhibition zone of ethanol extract Diameter (mm) (Mean ± S.D)	
		E.coli	S.aures
*Euphorbia robecchi*	25	9.33 ± 0.33	10.33 ± 0.00
	50	12.33 ± 0.33	11.33 ± 0.33
	100	14.67 ± 0.33	13.00 ± 0.00
*Aloe megalacantha*	25	10.67 ± 0.33	9.33 ± 0.33
	50	12.33 ± 0.33	11.33 ± 0.33
	100	16.33 ± 0.33	14.00 ± 0.00
*Opoiliacampestris*	25	6.67 ± 0.33	6.67 ± 0.33
	50	7.67 ± 0.33	7.33 ± 0.33
	100	9.33 ± 0.33	8.67 ± 0.33
Tetracycline	Sta.	22.00 ± 0.00	22.00 ± 0.00

Values are expressed as the mean of three replicates ± standard deviation.

The article "Ethnobotanical study of traditional medicinal plants in Kebridehar and Shekosh districts, Korahi zone, Somali Region, Ethiopia" was retracted in 2025. Reasons: lack of ethics approval or compliance; concerns about the welfare of human subjects.

### 4.10 Determination of MIC andMBC

To evaluate the extracts' effectiveness against the tested bacterial strains, the minimum inhibitory concentration (MIC) was utilized. The previous antibacterial assay, which used the agar-well diffusion method, was only conducted on organisms that showed a zone of inhibition and were susceptible to the plant extracts. The greatest antibacterial activity of all the plant extracts tested was found to be in *Aloe megalacantha*. *Aloe megalacantha* methanol extract has a 12.5 mg/m MIC against gram-positive *S. aureus* bacteria (Table 15). Another gram-negative bacterium, *E. coli*, was found to have a concentration of 12.5 mg/ml (Table 16).

**Table 15:** Gram-positive bacterial MICs and MBCs results.

		Methanol Extract (mg/ml)		Ethanol Extract (mg/ml)	
Plant Name	Bacteria Species	MIC	MBC	MIC	MBC
*Euphorbia robecchi*	*S.aureus*	25	50	30	60
*Aloe megalacantha*	*S.aureus*	12.5	25	25	50
*Opoiliacampestris*	*S.aureus*	75	150	100	200

Gram-Negative Bacterial MICs and MBCs Results.

**Table 16:** Gram-negative bacterial MICs and MBCs results.

		Methanol Extract (mg/ml)		Ethanol Extract (mg/ml)	
Plant Name	Bacteria Species	MIC	MBC	MIC	MBC
*Euphorbia robecchi*	*E.coli*	25	50	30	60
*Aloe megalacantha*	*E.coli*	12.5	25	25	50
*Opoiliacampestris*	*E.coli*	75	150	100	200

Gram-Positive Bacterial MICs and MBCs Results.

## 5 Discussion

### 5.1 Demographic status of knowledge

Elders and family members of the community have a concentration of ethnomedicinal knowledge, and passing it on to the younger generation is challenging. Most respondents (39.19 %) preferred the educational status of their native knowledge to their religious education, while the other respondents in grades eight through twelve (5.41 %) chose learning about medicinal plants. Poor indigenous knowledge transmission to the next generation is thought to be a factor in the practice's potential decline. The study found that modernization has an impact on how medicinal plant knowledge is transmitted to the next generation. This may be due to the younger generation's declining interest in indigenous knowledge. Similar findings on young people's lack of interest in conventional medicinal plants were reported by Ref. [12].

The article "Ethnobotanical study of traditional medicinal plants in Kebridehar and Shekosh districts, Korahi zone, Somali Region, Ethiopia" was retracted in 2025. Reasons: lack of ethics approval or compliance; concerns about the welfare of human subjects.

The number of species reported by the informants was positively correlated with their age. Younger people exhibited less interest in studying and using ethnomedical techniques, which may be related to their exposure to modern education. The fact that conventional knowledge is developed over many years of experience, according to Ref. [11], may explain why young people have less knowledge about medicine. The younger generation is quickly being drawn into a new tradition as a result of advances in science and technology. This study confirms the findings of [1], who found that younger generations have less knowledge than older ones.

### 5.2 Medicinal plants of the study area

In the study area, forty-four medicinal plants were reportedly used by local informants to treat both human and livestock ailments. These plants fall within the 34 genera and 23 family categories (Appendix 2, supplementary material). This result is clear evidence that the area under study is home to numerous plant species and kinds. Fabaceae led the way with 9 species (20.45 %), followed by Burseraceae, Euphorbiaceae, and Solanaceae with 4 each (9.09 %) and Tiliaceae, Cucurbitaceae, Lamiaceae, and Malvaceae with 2 each (4.54 %). The remaining families were represented by 1 species (2.27 %) (Fig. 2, Appendix 3, supplementary material).

Since the use of traditional medicinal herbs has been documented everywhere in Ethiopia, the locals of these places have a wealth of indigenous knowledge on the subject [13,14]. On the other hand, most indigenous knowledge gathered from the neighborhood is kept secret and passed down verbally among relatives. As a result, there is a chance that indigenous knowledge will be lost in the transfer system. Indigenous knowledge is at risk from modernization, untimely parent loss, religious authorities, and the public's perception of practitioners.

Although traditional medicine plays a significant role in the society of the study area, there are many misconceptions regarding its knowledge and practices, particularly among the younger generation and certain modern health professionals who dismiss it as if it were completely detrimental. On the other hand, traditional medicine is vital to the community since it serves as the only means of treatment for people who reside outside of the city, where there are few contemporary healthcare facilities.

### 5.3 Habits of medicinal plants

In the study area, not all plant growth forms are equally used as treatments. This is a result of the different growth type's distributions. As a result, plants are frequently employed for therapeutic purposes. This result implies that shrubs, followed by trees, are the most prevalent type of medicinal plant in the study area. In Ethiopia's Berbere District and Oromia region, similar results were also found [15]. In a more recent investigation [16], reported that shrubs were mostly used in the preparation of traditional remedies.

The article "Ethnobotanical study of traditional medicinal plants in Kebridehar and Shekosh districts, Korahi zone, Somali Region, Ethiopia" was retracted in 2025. Reasons: lack of ethics approval or compliance; concerns about the welfare of human subjects.

In contrast, this analysis contradicts the majority of Ethiopian inventories of medicinal plants [11,17], which indicate that herbs are the most prevalent kind of medicinal plant growth. This result may be the result of several environmental factors.

Medicinal Plants Used to Treat Human, Livestock, and Both Human and Livestock Ailments in the Study Area.

Plant species that are used to treat human ailments were discovered in the study area. These plants are divided into 22 families and 31 genera. Eight species came from the Fabaceae family, four from the Solanaceae, three each from the Burseraceae and Euphorbiaceae, two each from the Malvaceae and Tiliaceae, and one from each of the other ten families. Plant species used to alleviate livestock issues were noted in the study area. There are five genera and five families of such plants. Local inhabitants prioritized the use of medicinal herbs to cure human ailments rather than cattle diseases and sought out more indigenous knowledge. Similar results were discovered at additional Ethiopian research sites [18].

In another case, ailments in both humans and livestock are treated using the same species and component combinations. For instance, the glue of *Commiphoraguidotti* is the only species in the study area that is used to treat human stomach illnesses and to remove unwanted objects from livestock after delivery. As a result, the research area had a wide variety of indigenous knowledge regarding the use of medicinal plants to treat various illnesses.

Parts of Medicinal Plants Used to Treat Human and Livestock Ailments.

Parts of medicinal plants are used to treat human ailments.

The roots of plants were the plant parts that were most frequently utilized to make medicines. The fact that roots are chosen above other plant parts for disease therapy may be due their chemical composition of roots. Remedy formulations involving roots, rhizomes, bulbs, barks, stems, or the entire plant have effects that pose a longer-term harm to the plant's life in comparison to leaf preparations.

While roots were the most commonly collected plant part in the area and had a substantial impact on the mother plant's survival, this research region's medicinal plants are most at risk from plant parts used for medical purposes. The discovery that roots account for a greater proportion of plant species used for medicinal purposes than other plant parts is consistent with a study conducted by Ref. [19], in which roots (31.4 %) were found to be the most commonly utilized plant component, followed by leaves (24.4 %). According to the [15] study, roots account for 42 % of all plant components used. In addition, root (35.8 %) was listed as a significant plant component used in the treatment of human illnesses [10]. According to a study by Ref. [15], 44.8 % of plants used to treat human illnesses have roots.

The article "Ethnobotanical study of traditional medicinal plants in Kebridehar and Shekosh districts, Korahi zone, Somali Region, Ethiopia" was retracted in 2025. Reasons: lack of ethics approval or compliance; concerns about the welfare of human subjects.

This finding contradicts those of other ethnomedical studies. The most utilized plant part in curative compositions, according to Refs. [11,20], and [15], is the leaf. This variation suggests that the mother plant might be impacted by diverse environmental factors and root systems. However, according to Refs. [15,20] studies, leaves are primarily used in traditional medicinal formulations. The harvesting of leaves could be marketed as a more sustainable method because, in most cases, at least many leaves are left over on the parent plant and because it has been reported that medicinal plant species' leaves are also harvested for most cure preparations alongside roots.

### 5.4 Mode of preparation used to treat human and livestock ailments

#### 5.4.1 Mode of preparation used to treat human ailments

According to studies, Ethiopians have long used conventional medicinal plants as treatments [5,14]. The local community employs a number of techniques to create traditional medicines for a variety of conditions while preparing medication for humans. Depending on the ailment being treated and the location of the issue, several preparations are used. The informants are skilled in many different areas of medicine preparation. In their work, they typically make use of various plants. According to Refs. [12,15], who indicated that crushing was the primary way of remedy preparation, crushing is the second most common mode of preparation in the study area. Crushing powder is the primary mode of preparation in the study area [10].It was revealed that powdering was the predominant method of medicine production in a survey of residents of the Wonago District. According to the research, the majority of medicines were created from a single plant species and used to treat a disease. The results concur with those of [21], who discovered a high yield from a single plant preparation. *Commiphoraguidottii* is the only species that can be used to treat both human and cattle ailments.

Some of the additives utilized in various treatments include water, boiled coffee, tea, butter, salt, milk, and others. Informants report that these substances are essential for reducing discomfort, enhancing efficacy, improving flavor, minimizing unpleasant consequences, including vomiting and diarrhea, and improving healing conditions. A straightforward and effective treatment method can involve combining medicinal herbs with common foods and drinks. *Belpharisedulis*, for instance, can be extracted by crushing the plant's middle section and boiling it with milk or tea to drink, or by cooking it with meat to consume. A patient is advised to try this as a stomach remedy.

The article "Ethnobotanical study of traditional medicinal plants in Kebridehar and Shekosh districts, Korahi zone, Somali Region, Ethiopia" was retracted in 2025. Reasons: lack of ethics approval or compliance; concerns about the welfare of human subjects.

#### 5.4.2 Mode of administration human and livestock ailments

The conclusion of this study is that the mode of administration in human ailments has the highest value of the oral delivery method found, and this result is in line with other Ethiopian investigations [1,2], and [5]. The dermal administration method is the leading method to treat livestock ailments in the study area.

## 6 Ranking of important medicinal plants

### 6.1 Preference ranking

The most effective medicinal plant to treat ulcers is *Euphorbia robecchii*, which came in first place in a preference rating of six ulcer-treating plants. The second, third, fourth, and fifth most desired therapeutic herbs against this condition, respectively, are *Grewiatenax, Hydnorajohannis, Lyciumshawii*, and *Ricinuscommunis*, whereas *Desmodiummolliculum* is the least preferred out of the six species, according to informants.

*Euphorbia robecchii* earned the highest mark and placed first, suggesting that it was the most beneficial in curing ulcers. It was followed by *Grawiatenax* in the results (Table 5). In the other most prevalent disorder, stomachache was cured by an herbal remedy, *Stephania abyssinica,* as reported by Ref. [15] in other areas of Berbere district in the Oromia region.

### 6.2 Paired comparison

Five medicinal plants were compared by six key informants in pairs, and the outcomes were compiled. Gastrointestinal ulcers can be successfully treated using *Acacia senegal* species, *Aloe megalacantha*, *Moringastenopetala*, and *Commiphoraguidottii*. The least-favorable species for treating the illness in the region was *Blepharisedulis*. This rating, at least from the perspective of locals, is a result of the plant's effectiveness (Table 6). In the other study location [15], it was observed that *Oleaeuropaea*medicinal plants were extensively used to treat wounds in different areas of the Berbere district and Oromia region.

### 6.3 Informant consensus

In the study area, some of the species were well-known and regarded as top treatments. Examples include *Grrewia species*, *Solaniumincanum*, *Euphorbia schizocantha*, *Commiphoragudidotti*, *Commiphoramyrra*, and *Moringastenopetala* (Table 8). Due to the abundance of the species and the nature of the ailments they treated, these medicinal plants were well known and widely used.

The article "Ethnobotanical study of traditional medicinal plants in Kebridehar and Shekosh districts, Korahi zone, Somali Region, Ethiopia" was retracted in 2025. Reasons: lack of ethics approval or compliance; concerns about the welfare of human subjects.

### 6.4 Informant consensus factor (ICF)

The results show that frequent diseases in the study area have a higher informant consensus factor. Moreover, medicinal plants with higher ICF values (Table 9) and ICF values ranging from 0.88 to 0.67 for each disease category are well known by locals and effective in treating particular disorders. The ICF values for cancer, fertility, and maternity were the lowest (0.67), due to their rarity and the fact that the majority of cases are successfully treated by local healers. Malaria and fever had the highest ICF values (0.88) because of the high prevalence of the disorders in the area. The results showed that local people used ethnomedicinal plants in a number of different ways to treat illnesses. One kind of plant is used to cure two or more diseases. Many plants, including *Adeniumsomalense*, *Belpharisedulis,* and *Azadirachtaindica*, have been utilized to cure a variety of illnesses. The same type of illness is treated with a variety of plant species.

### 6.5 Jaccard coefficient of similarity

The two people most like each other are the southwest Oromo and this study. The socio-cultural elements that affect people's awareness of medicinal plants are most likely to blame for this. The relative proximity of the research areas may also increase the amount of cultural input. The least similarity is found in WonagoWereda, which may be explained by the two research locations' different vegetation patterns and the two populations' various cultural traditions.

### 6.6 Threats from medicinal plants in the study area

#### 6.6.1 Factors threatening medicinal plants

Medicinal plants are increasingly in danger due to habitat degradation (agricultural expansion, fire, construction, overgrazing, and urbanization) and overharvesting of species recognized to be beneficial [5,15]. According to Ref. [22], one significant medicine candidate disappears from the planet every two years, and 15,000 medicinal plant species may be globally in danger of extinction as a result of habitat loss and overharvesting. Firewood was identified as the top threat to medicinal plants in the research area, with drought coming in second. According to Ref. [14] findings, the main danger to Zay people's access to medicinal plants was severe deforestation. The majority of Ethiopians use traditional medicine as their primary form of healthcare. Two types of risks exist for medicinal plants: those brought on by nature and those imposed by people. However, in addition to natural factors, anthropogenic factors like deforestation due to overexploitation of plants for various uses like the production of charcoal, the collection of firewood, the gathering of wood for construction, and overgrazing are reported in this study as threats to medicinal plants and related indigenous knowledge. According to the informant, firewood is the greatest threat to medicinal plants, followed by drought and charcoal harvesting, while overgrazing poses a less serious threat (Table 12). According to local environmental considerations, anthropogenic factors differ by place. Risks to medicinal plants in Wonago District include agricultural expansion (24.4 %), firewood collection, and others, according to Ref. [10]. Moreover [14], made a point about how deforestation harms medicinal plants. According to the present research area's findings, firewood was the most crucial element, which is consistent with earlier studies [16]. [12] Reported that the biggest threats to the medicinal plants in the Sekoru district of the Jimma zone were deforestation (40 %) and agricultural expansion (12.5 %).

The article "Ethnobotanical study of traditional medicinal plants in Kebridehar and Shekosh districts, Korahi zone, Somali Region, Ethiopia" was retracted in 2025. Reasons: lack of ethics approval or compliance; concerns about the welfare of human subjects.

As a result of their widespread exploitation for uses other than medicine, it is clear that proper consideration for their conservation is necessary. Due to agricultural development, deforestation, fire, overgrazing, charcoal and firewood production, and other factors, the amount of natural vegetation has drastically decreased, which has had an impact on the availability of medicinal plants [15]. The challenges for the preservation of medicinal plants and related information are caused by human influences on the natural habitat of medicinal plants. It was found that very little was being done in the district to preserve medicinal plants. Although the effort was small, some individuals have begun to conserve medicinal plants by cultivating them in backyard gardens.

Natural resources could be used most effectively and sustainably if management practices are thorough, according to a suggestion made by Ref. [23]. The full range of societies and stakeholders involved in the preservation, production, management, and use of medicinal plants are actually required to take the proper actions and make the necessary changes in order to continue these worthwhile endeavors. It is necessary to continuously work on raising public awareness because efforts to conserve and use medicinal plants sustainably require the involvement of various sectors and greater public support [24].

#### 6.6.2 Activities on gram-negative and gram-positive bacteria

Antibiotic resistance is a subject that continues to pose difficulties for the healthcare industry in both developed and developing nations throughout much of the world. The existing antibiotic therapy is significantly threatened by the emergence and spread of multidrug-resistant organisms. Since plants contain a variety of bioactive chemicals with proven medicinal capabilities, the quest for new sources of antibacterial agents has been necessary. This research was done to assess the antibacterial activity of various medicinal plant extracts against two reference strains of human infections [25].

The article "Ethnobotanical study of traditional medicinal plants in Kebridehar and Shekosh districts, Korahi zone, Somali Region, Ethiopia" was retracted in 2025. Reasons: lack of ethics approval or compliance; concerns about the welfare of human subjects.

The antibacterial activity of several plant extracts against the test bacterial isolates was restricted, as shown by their MIC values, despite the fact that some extracts showed good antibacterial activity against various tested bacterial isolates. The results showed that, among the investigated gram-negative organisms, *E. coli* clinical isolates were the most susceptible bacteria. *E. coli* gram-negative bacteria were sensitive to both methanol and ethanol extracts at 100 mg/ml, with inhibitory zones spanning from 9.33 ± 0.33 to 20.00 ± 0.00 and 9.33 ± 0.33 to 16.33 ± 0.33 mm, respectively (Table 13, Table 14).

The most effective against *S. aureus* and *E. coli* at a concentration of 100 mg/ml was *Aloe megalacantha* root extract, followed by *Euphorbia robecchi.Aloe megalacantha* extracts demonstrated the most potent anti-*E. coli* activity when compared to typical antibiotics found in tetracycline. *Aloe megalacantha*and *Euphorbia robecchi* extracts showed statistically significant inhibition of *E. coli* in the study area at doses of 50 and 100 mg/ml, respectively. In accordance with [26], Aloe species of *Aloe adigratana* inhibited *S.aureus* at 200 mg/ml 16.63 ± 0.12.

In our tests, we found that Tetracycline was effective against *E. coli* and *S. aureus* at a standard concentration of 22.00 mm. The chosen plant extracts demonstrated noticeably higher inhibitory activity at 100 mg/ml compared to 50 mg/ml in the tested gram-negative bacterial species in both methanol and ethanol extracts.

### 6.7 Determination of MIC and MBC

Gram-Positive Bacterial MICs and MBCs Results.

Gram-positive bacterial strains were exposed to various concentrations of plant extracts to test *S. aureus* antibacterial abilities. The MIC, or minimum inhibitory concentration, was then calculated using an agar dilution assay. The MIC is defined as the lowest concentration of an antibacterial agent that inhibits bacterial growth after 24 h at 37° Celsius. In accordance with [26], Aloe species of *Aloe adigratana* are the most potent compounds against *S. aureus* with 0.06 ± 0.025.

Table 15 shows that *Aloe megalacantha* methanol extracts had high action against the bacteria tested, with a MIC of 12.5 mg/ml, followed by *Euphorbia robecchi* methanol extract, which had a MIC of 25 mg/ml. *S. aureus,* with a concentration of 12.5 mg/ml, was the most vulnerable bacteria in the treatment with *Aloe megalacantha* methanol extracts. *Aloe megalacantha* with methanol extract demonstrated possibly bactericidal action against tested gram-positive bacteria, with an MBC of 25 mg/ml against *S. aureus* and *Euphorbia robecchi*at 50 mg/ml against *S. aureus.*

The article "Ethnobotanical study of traditional medicinal plants in Kebridehar and Shekosh districts, Korahi zone, Somali Region, Ethiopia" was retracted in 2025. Reasons: lack of ethics approval or compliance; concerns about the welfare of human subjects.

Gram-Negative Bacterial MICs and MBCs Results.

Agar dilution was employed to further assess the antibacterial properties of *E. coli* with methanol and ethanol extract against gram-negative bacterial species using quantitative methodologies, and MIC and MBC were determined as shown in Table 16. *Aloe megalacantha* methanol extract showed the lowest antibacterial potential for *E. coli* with a 12.5 mg/ml MIC value, followed by *Euphorbia robecchi* with a 25 mg/ml MIC value. The ethanol extract of *Aloe megalacanta*, on the other hand, showed the lowest potential antibacterial activity against *E. coli*, with a MIC of 25 mg/ml and an MBC of 50 mg/ml.

## 7 Conclusion and recommendation

In the research region, a large number of therapeutic plants were discovered. It was also demonstrated that traditional medicinal plants are extremely important and that the local community has extensive indigenous medicinal knowledge to aid with the District's primary healthcare needs (for both humans and animals). Malaria, fever, hemorrhoid, cardiovascular disease, diarrhea, typhoid, ulcers, skin illnesses, and stomach and gastric ailments are some of the diseases that traditional healers in the area choose to cure. Secrecy, oral-based information transfer, the unwillingness of young generations to obtain knowledge, the unavailability of species, the effect of contemporary education, and awareness issues are among the greatest threats to indigenous knowledge.

Our findings revealed that *Aloe megalacantha* was the most powerful of the therapeutic plants tested. Following the isolation and identification of active compounds from the plants, which can serve as leading compounds in antibacterial drug development for the treatment of bacterial origins, these plants may be the ideal choice for further studies in the creation of new antibacterial agents. Encourage people to grow medicinal plants in their backyard gardens. Encourage local herbal medicine practitioners to use traditional medicine more effectively by providing licensure and other incentives, as well as encouraging local people to participate in conservation programs.

## Data availability

The dataset used to support the findings of this study is included within the text and supplementary materials.

The article "Ethnobotanical study of traditional medicinal plants in Kebridehar and Shekosh districts, Korahi zone, Somali Region, Ethiopia" was retracted in 2025. Reasons: lack of ethics approval or compliance; concerns about the welfare of human subjects.

## Funding

Not applicable.

## Declaration of competing interest

The authors declare that they have no known competing financial interests or personal relationships that could have appeared to influence the work reported in this paper.
